The article "Glycol chitosan incorporated retinoic acid chlorochalcone (RACC) nanoparticles in the treatment of Osteosarcoma" was retracted in 2020. Reasons: results that could not be reproduced; duplicated images; concerns about the images.

# Glycol chitosan incorporated retinoic acid chlorochalcone (RACC) nanoparticles in the treatment of Osteosarcoma

**DOI:** 10.1186/s12944-015-0068-4

**Published:** 2015-07-14

**Authors:** Yan-Guo Qin, Lan-Yu Zhu, Chen-Yu Wang, Bo-Yan Zhang, Qing-Yu Wang, Rui-Yan Li, Zhen Liu

**Affiliations:** Department of Orthopedics, The Second Hospital of Jilin University, Changchun, Jilin 130041 China; Nursing School, Changchun University of Chinese Medicine, Changchun, Jilin 130117 China; Norman Bethune Medical School, Jilin University, Changchun, Jilin 130021 China

**Keywords:** Osteosarcoma, Membrane potential, Migration, Inhibition, Glycol chitosan

## Abstract

**Background:**

Osteosarcoma is the most common of all the bone malignancies and accounts for 30-80 % of the primary skeletal sarcomas. The overall survival rate of patients with osteosarcoma is < 20 % suggesting poor prognosis.

**Methods:**

The present study demonstrates the effect of retinoic acid chlorochalcone (RACC) incorporated glycol chitosan (GC) nanoparticle transfection in osteosarcoma cells. MG-63 and Saos-2 osteosarcoma cells were transfected with various concentrations of RACC-incorporated GC nanoparticle for 24 h. The effect on cell proliferation, Ezh2 expression, apoptosis, cell cycle arrest, cell migration and invasiveness, Akt phosphorylation and local tumour growth and metastases were studied.

**Results:**

MG-63 and Saos-2 osteosarcoma cells on RACC-incorporated GC nanoparticle transfection for 24 h showed a concentration-dependent inhibition of cell proliferation. Of the various concentrations of RACC tested, the effective concentration started from 5 μM with an IC_50_ of 20 μM. Wound healing assay also showed that RACC-incorporated GC nanoparticles inhibited migration of tumor cells more effectively compared to the parent RA. RACC transfection resulted in inhibition of cell proliferation, Ezh2 expression inhibition, apoptosis through mitochondrial pathway by decrease in membrane potential and release of cytochrome c and cell cycle arrest in the G0/G1 phase. The invasiveness of cells treated with 5 and 20 μM RACC was decreased by 49 and 76 % respectively, compared to the control. RACC-treated mice showed significantly lower number of metastases compared to that in the control mice.

**Conclusions:**

Thus, RACC-incorporated glycol chitosan nanoparticle strategy can be promising for the treatment of osteosarcoma.

## Background

Osteosarcoma is the most common of all the bone malignancies and accounts for 30-80 % of the primary skeletal sarcomas [1, 2]. It frequently attacks the children, teenagers, and young adults between 10–30 years of age [3]. Compared to females osteosarcoma is more predominantly observed in males. The long cylindrical bones like femur, tibia, and humerus including the knee joint are the main target in osteosarcomas [4]. However, the shoulder blade, pelvic, and skull bones are also sometimes affected [5]. Osteosarcoma is a well-defined clinical entity with a characteristic radiographic appearance, histologic features, a relatively consistent spectrum of clinical presentations, and established standard treatments. These features have been the subject of many prior book chapters and reviews [6–11]. However, all of the present treatments are less efficient. Therefore, the discovery of molecules with roles in the osteosarcoma inhibition is highly desired to improve the clinical treatment.

The article "Glycol chitosan incorporated retinoic acid chlorochalcone (RACC) nanoparticles in the treatment of Osteosarcoma" was retracted in 2020. Reasons: results that could not be reproduced; duplicated images; concerns about the images.

Polycomb group of genes (PcG) which play a crucial role epigenetically in regulating gene transcription programs possess a catalytic subunit, Enhancer of Zeste homolog 2 (Ezh2) [12]. It has been demonstrated that Ezh2 controls expansion and differentiation of tumor initiating cells and the development and progression of cancer [13–15]. In Myelodysplastic syndromes Ezh2 functions as a tumor suppressor [16, 17]. It inhibits cell differentiation to maintain stemness of tumor cells [18, 19].

Retinoic acids (RAs) have been used in the prevention and treatment of dermatological diseases [20, 21]. Recently retinoic acid and other retinoids have been reported to possess promising anti-cancer activity [22]. It was demonstrated that retinoic acids affect in vitro proliferation, differentiation, and apoptosis of colon [23], prostate [24], lung [25], and leukemia [26] cancers. Moreover, retinoc acids also influence the morphological differentiation, proliferation, and gene expression of neuroblastoma [27] and astrocytoma cells [28]. Recurrent malignant cerebral gliomas have been treated with ATRA [29, 30] and 13-*cis* RA [31]. Despite of its in vitro biological promise, its poor bioavailability under in vivo restricts its clinical applications [32]. One of the techniques to overcome this drawback is the development of polymeric micelles [33], like glycol chitosan micelle. Taking cue from the above literature we devised an experiment to study the effect of RACC (Fig. 1) having more bioavailability compared to the parent compound on human glioma.

**Fig. 1:** Structure of retinoic acid chlorochalcone (RACC) and glycol chitosan (GC)

## Results

### RACC-incorporated GC nanoparticles cause proliferation inhibition in human osteosarcoma cells

The results from MTT assay revealed a dose-dependent inhibition of the MG-63 and Saos-2 cell proliferation on RACC treatment after 24 h. Among the range of concentrations from 1 to 20 μM tested, the inhibition was significant at 5 μM with a reduction in O.D. values of 16 ± 0.6 and 13 ± 0.8 % for MG-63 and Saos-2 cell lines respectively. The reduction in O.D. values at 10, 15 and 20 μM was 23 ± 2, 63 ± 3.5, 90 ± 10 % for MG-63 and 36 ± 3.2, 64 ± 3.43 and 89 ± 10.34 for Saos-2 cells respectively. The IC_50_ values of RACC were 18.2 ± 2.8 μM for both the tested cell lines.

The article "Glycol chitosan incorporated retinoic acid chlorochalcone (RACC) nanoparticles in the treatment of Osteosarcoma" was retracted in 2020. Reasons: results that could not be reproduced; duplicated images; concerns about the images.

The daily MTT assay using 20 μM RACC for 4 days showed that growth inhibition for both the cell lines was maximum at day 4 (Fig. 2a,c). The trypan blue exclusion assay showed drop in cell number in a time-dependent manner (Fig. 2b,d).

**Fig. 2:** RACC-incorporated GC nanoparticles induced time-dependent inhibition of MG-63 and Saos-2 cell proliferation. **a** and **c**, MTT tests on MG-63 and Saos-2 osteosarcoma cell line; **b** and **d**, trypan blue tests on MG-63 and Saos-2 osteosarcoma cell line. Cells were cultured in medium containing empty GC vesicles (□) or RACC-incorporated GC nanoparticles (●) with 20 μM RACC, added at a day “0,” for the time indicated. Results correspond to three different experiments and values are expressed as mean

### RACC-incorporated GC nanoparticle transfection inhibits Ezh2 expression in human osteosarcoma cells

We used Western blot and RT-PCR analysis to examine the changes in Ezh2 and protein expression levels in MG-63 and Saos-2 cells on RACC-incorporated GC nanoparticle treatment. The results showed a significant decrease in Ezh2 expression level after 24 h of RACC-incorporated GC nanoparticles (20 μM) transfection compared to control. The Ezh2 inhibition by RACC lasted for at least 72 h after the RACC-incorporated GC nanoparticle transfection (Fig. 3). These results suggest that after the transfection of the RACC at 20 μM for 24 h, the Ezh2 and protein expression levels are effectively inhibited.

**Fig. 3:** Expression of Ezh2 and protein in MG-63 and Saos-2 cells after RACC transfection. **a** and **c** After the MG-63 and Saos-2 cells were transfected with 20 μM RACC, the expression level of the Ezh2 and proteins was significantly reduced. **b** The efficacy of RACC to inhibit the Ezh2 expression was further analysed by western blotting analysis

### RACC-incorporated GC nanoparticles induce apoptosis in MG-63 and Saos-2 human osteosarcoma cells

We used flow-cytometric and ssDNA detection assay to examine apoptotic cell death in osteosarcoma cells. In MG-63 cells treatment with 5 and 20 μM RACC induced apoptosis in 5.89 ± 3.9 and 60.54 ± 5.4 % cells respectively compared to 2.05 ± 1.01 % cells in control (Fig. 4). Similar results were observed in Saos-2 cells, where in exposure to 5 and 20 μM RACC induced apoptosis in 9.86 % ± 8.89 and 47.54 ± 14.5 cells respectively compared to 1.79 ± 0.23 % in control cells (data not shown).

The article "Glycol chitosan incorporated retinoic acid chlorochalcone (RACC) nanoparticles in the treatment of Osteosarcoma" was retracted in 2020. Reasons: results that could not be reproduced; duplicated images; concerns about the images.

**Fig. 4:** RACC-induced apoptosis in MG-63 cells. Cultures were grown either in medium containing empty GC vesicles (control) or in a medium containing 5 μM or 20 μM RACC. The arrows indicate apoptotic cells; magnified image of cells was shown in corner

### RACC treatment induces apoptosis in the MG-63 and Saos-2 human osteosarcoma cells through the mitochondrial pathway

We used JC-1 staining to detect the changes in mitochondrial membrane potential in MG-63 and Saos-2 cell lines. The results clearly showed that increase in concentration of RACC in RACC-incorporated GC nanoparticle from 10 μM to 25 μM significantly reduced the mitochondrial membrane potential in MG-63 cells (Fig. 5a). Western blot analysis revealed translocation of Bax and Bcl-2 proteins from mitochondria to cell cytosol (Fig. 5b). Similar results were obtained in Saos-2 human osteosarcoma cell lines.

**Fig. 5:** RACC induces apoptosis in MG-63 cells through the mitochondrial pathway. **a** Changes in the mitochondrial membrane potential were analysed by JC-1 staining and subsequent flow cytometry. **b** The expression levels of Bax, Bcl-2, and cytochrome c in the cytoplasm and mitochondria were analysed by western blotting

### RACC-incorporated GC nanoparticle transfection causes a cell cycle arrest in the G0/G1 phase in MG-63 and Saos-2 human osteosarcoma cells

The results from flow cytometry showed a significant increase in G0/G1 cell population in both MG-63 and Saos-2 cells with subsequent decrease in S and G2/M phase on treatment with RACC (5 μM) (Fig. 6). The increase in concentration of RACC from 5 μM to 20 μM led to further increase in the percentage of cells in G0/G1 phase and subsequent decrease in cell percentage from S and G2/M phase (Fig. 6). These results confirm that RACC transfection arrests cell cycle in G0/G1 phase in human osteosarcoma cell lines.

**Fig. 6:** Effect of RACC transfection on cell cycle arrest in MG-63 and Saos-2 cells. The cell cycle distribution of MG-63 and Saos-2 cells that had been treated with empty GC vesicles. The cell cycle distribution of MG-63 and Saos-2 cells that had been treated with 5 and 20 μM RACC incorporated GC nanoparticles

### RACC-incorporated GC nanoparticle transfection inhibits cell migration and invasiveness

Treatment with RACC (20 μM) for 24 h significantly decreased the migratory activity of MG-63 and Saos-2 cells by 52 and 58 % respectively compared to control cells (Fig. 7a). The migratory activity of the cells treated with 5 μM RACC was decreased by 10 and 40 % respectively in MG-63 and Saos-2 cells. In invasion assay, the capacity of the RACC-treated MG-63 cells to pass though the Matrigel-coated filters was significantly lower compared to control cells (Fig. 7b). The invasiveness of cells treated with 5 and 20 μM RACC was decreased by 49 % and 76 % (P < 0.001), respectively, compared to the control. Knockdown of Has1 and/or Has3 with siRNA revealed that the single knockdown of Has1 or Has3 did not compensate for the effects of RACC on cell motility or invasiveness, however the double knockdown of Has1 and Has3 did (Fig. 7c). Thus suggesting the involvement of HA-dependent route in the inhibitory effects of RACC on cell motility and invasiveness.

The article "Glycol chitosan incorporated retinoic acid chlorochalcone (RACC) nanoparticles in the treatment of Osteosarcoma" was retracted in 2020. Reasons: results that could not be reproduced; duplicated images; concerns about the images.

**Fig. 7:** Effect of RACC on cell motility, invasiveness, and Akt-phosphorylation. **a** Cell motility of MG-63 and Saos-2 cells. **b** Cell invasiveness of MG-63 cells. The number of cells on the lower surface of the membrane was counted in 20 randomly selected high-power fields. The data are presented as the average ± s.d. compared with DMSO). **c** Cell motility and invasiveness of MG-63 cells after knockdown of Has1 and/or Has3. The data are presented as the average ± s.d. compared with DMSO). **d** Western blotting for Akt phosphorylation

### RACC-incorporated GC nanoparticle transfection inhibits Akt phosphorylation

We also examined the effect of RACC treatment on Akt phosphorylation in MG-63 and Saos-2 cells using western blot analysis. The results revealed a significant decrease in Akt phosphorylation after 5 and 10 h of RACC treatment than that in the control cells. However, no difference was observed at 1 or 2 h (Fig. 7d).

### RACC-incorporated GC nanoparticle transfection exhibits inhibitory effects on local tumour growth and metastases

Administration of 20 μM RACC exhibited an inhibitory effect on MG-63 tumour growth, based on the reduction in tumour wet weight (67 % reduction, Fig. 8a). We used HABP staining to analyse the HA retention in the local tumour inhibited by RACC treatment. The results revealed a significantly lower HA retention in RACC-treated local tumours compared to that in the control tumours (Fig. 8c-e). RACC treatment resulted in a significant (84 %) reduction in the number of metastatic lesions which was visually analysed (Fig. 8b). RACC-treated mice showed significantly lower number of metastases compared to that in the control mice.

**Fig. 8:** Effect of RACC on implanted tumour mass and osteosarcoma metastasis of MG-63 cells. **a** The wet weights of the transplanted tumour were measured. (**b**) The numbers of osteosarcoma metastases. Representative sections of transplanted tumours with HABP staining (**c** and **e**; Control, **d** and **f**; RACC treatment)

## Discussion

In the present study, RACC-incorporated GC nanoparticles formed by electrostatic interaction between –COOH group of RACC and –NH_2_ group of glycol chitosan were prepared. The presence of reactive –NH_2_ group makes chitosan a suitable substrate for drug conjugation and ion complex formation with anionic drugs [14, 34–36]. Thünemann and Beyermann initially developed the concept of nanoparticle formation acid and positively charged macromolecules [29, 30]. Since then nanoparticle targeted treatment of cancer has been studied extensively [31–33].

The article "Glycol chitosan incorporated retinoic acid chlorochalcone (RACC) nanoparticles in the treatment of Osteosarcoma" was retracted in 2020. Reasons: results that could not be reproduced; duplicated images; concerns about the images.

Taking into consideration poor bioavailability of RACC, we transfected RACC-incorporated GC nanoparticles into human osteosarcoma cells to investigate its effect on cell proliferation and cell cycle. There was significant inhibition in cell proliferation on treatment with RACC-incorporated GC nanoparticles at a concentration of 20 μM of RACC within 24 h. The proliferation inhibition continued for 72 h and the effect was seen to be maximum on day 4. Further investigation revealed that RACC transfection in MG-63 and Saos-2 human osteosarcoma cells caused inhibition of Ezh2 expression. The inhibition was seen after 24 h of RACC transfection at 20 μM (IC_50_ value) concentration and lasted for 72 h. The results from apoptosis and necrosis assay showed increase in the percentage of apoptosis on increasing the concentration of RACC. Our results from flow-cytometry demonstrate that osteosarcoma cells undergo apoptosis through mitochondrial pathway. The Bax and Bcl-2 proteins were seen to translocate from mitochondria into cytoplasm where they led to release of cytochrome c. Cytochrome c then activates caspase 9 and caspase 3, which play key roles in the apoptosis pathway [37]. The increase in concentration of RACC in RACC-incorporated GC nanoparticle from 5 μM to 20 μM significantly reduced the mitochondrial membrane potential in MG-63 cells. Therefore, these results suggest that the RACC inhibition of Ezh2 expression induces apoptosis through the mitochondrial pathway in human osteosarcoma cells. Our results from flow cytometry also suggest that RACC induces cell cycle arrest in G0/G1 phase. Treatment of MG-63 and Saos-2 cells with 10 μM concentration of RACC, led to an increase in the percentage of cells in G0/G1 phase with the subsequent decrease in S and G2/M phase. The increase in concentration of RACC from 5 μM to 20 μM significantly increased the percentage of cells in G0/G1 phase.

The results from our study revealed that RACC exerted a multistep inhibitory effect on the tumourigenicity of osteosarcoma cells through inhibition of HA synthesis. HA being the major component of ECM, the reduction of Has subsequently causes the suppression of ECM production, particularly that of the cell-associated matrix. It is reported that cell-associated matrix is linked to tumourigenicity [38–40]. Our results demonstrate that the inhibition of cell-associated matrix formation through suppression of HA synthesis by RACC effectively suppressed the tumourigenicity. Thus, the anti-tumour activity of RACC may be partly through the depletion of cell-associated matrix formation.

The article "Glycol chitosan incorporated retinoic acid chlorochalcone (RACC) nanoparticles in the treatment of Osteosarcoma" was retracted in 2020. Reasons: results that could not be reproduced; duplicated images; concerns about the images.

Recent studies have shown that the PI3K/Akt signalling pathway is significantly involved in HA-induced cell motility and invasiveness. We also demonstrated that RACC-induced downregulation of Akt phosphorylation in osteosarcoma cells. Considering the delayed inhibition of Akt phosphorylation (after 6 h) by RACC in this study, RACC may indirectly affect Akt phosphorylation, possibly via suppression of HA synthesis, perturbation of HA-receptor interaction, or alteration of cell signalling pathways including Akt phosphorylation.

The degree of the inhibitory effects of RACC on the formation of osteosarcoma metastasis in vivo was markedly higher than that on the growth of the implanted primary tumour. In contrast to the growth of the primary tumour, multistep processes are associated with distant metastasis. In this study, RACC suppressed proliferation, motility, and invasion of osteosarcoma cells in vitro. Inhibition of these steps by RACC led to substantial suppression of tumour metastasis. Another explanation is that RACC affects the microenvironment of the primary and target organs. The tumour stroma and surrounding normal cells (immune cells, inflammatory cells, pericytes, vascular endothelial cells, and fibroblasts) can be affected by RACC, possibly via suppression of HA synthesis. Notably, in the current study, HA deposits were markedly suppressed not only in the periphery of the tumour, but also in the surrounding stromal tissues and perivascular region in vivo. In the clinical context, the strong suppressive effects of RACC on lung metastasis might be especially beneficial for patients with osteosarcoma, considering that the primary cause of death in this group is metastasis [41].

## Conclusions

The present study demonstrates that RACC inhibits various processes of tumourigenicity in vitro in murine and human osteosarcoma cell lines, and markedly suppressed osteosarcoma metastasis. Thus RACC-incorporated GC nanoparticles may be a promising strategy for the treatment of osteosarcoma.

## Materials and methods

### Cell culture

Human osteosarcoma cell lines, MG-63 and Saos-2 were purchased from the Health Science Research Resources Bank (Osaka, Japan). The cells were maintained in RPMI 1640 medium (RPMI:ECM = 4:1) supplemented with 10 % fetal bovine serum at 37 °C in 5 % CO_2_ in a humidified atmosphere.

The article "Glycol chitosan incorporated retinoic acid chlorochalcone (RACC) nanoparticles in the treatment of Osteosarcoma" was retracted in 2020. Reasons: results that could not be reproduced; duplicated images; concerns about the images.

### Chemicals and reagents

Glycol chitosan (GC), retinoic acid chlorochalcone (RACC), dialysis membranes (MWCO = 12,000 g/mol) and propidium iodide (PI) were purchased from Sigma Chem. Co. Ltd. (St. Louis, MO, USA). FITC-annexin V was obtained from Santa Cruz, CA, 95060, USA.

### Ethical statement

The present study was approved by the Institutional Review Board and Ethics Committee of the Nanjing University, Jiangsu, China.

### Preparation of RA-incorporated GC nanoparticles

The RACC-incorporated GC nanoparticles were prepared by adding a solution containing 5 mg RACC in 1 mL of DMF to an aqueous solution containing 40 mg of GC in 10 mL of deionized water while stirring. The stirring was continued for 20 min under darkened conditions. A dialysis membrane (MWCO = 12,000 g/mol, Sigma Chem. Co. Ltd. St. Louis, MO, USA) was used to prepare dialyzed solution against deionized water by dialysis for 1 day. Out of 20 mL prepared by adding deionized water to the dialyzed solution, 100 μL was diluted with 9.9 mL of DMSO. UV spectrophotometer (UV-1200, Shimadzu Co. Ltd., Kyoto, Japan) was used to measure drug contents at 365 nm and empty GC vehicles were used as a blank test.

### Proliferation inhibition assay (MTT assay)

In each well of a 96-well plate, aliquots containing 2.5 × 10^5^ cells were seeded. The cells were incubated overnight in a 5 % CO_2_ incubator at 37 °C and then RACC-incorporated GC nanoparticle solution was added to each well. After dilution with RIMI 1640 (10 % FBS), these were used to treat the tumor cells. RIMI 1640 (10 % FBS) with 0.1 % (v/v) DMSO was used as control. The incubation for 48 h was followed by addition of 25 μL of MTT (3 mg/mL in PBS) to each well and incubation was continued for 4 h more. To each well was added 100 μL of SDS–HCl solution (SDS 10 % w/v, 0.01 M HCl) and incubated again for 12 h. An Infinite M200 pro reader (Tecan Austria GmbH, Salzburg, Austria) was used to measure the absorbance at 570 nm. The viable cells were expressed as percentage of control and all the experiments were conducted in triplicate.

### Western blotting

The transfected osteosarcoma cells from were washed twice in PBS followed by addition of Lysis buffer (50 mM Tris–HCl pH 7.4, 137 mM NaCl, 10 % glycerol, 100 mM sodium vanadate, 1 mM PMSF, 10 mg/ml aprotinin, 10 mg/ml leupeptin, 1 % NP-40, and 5 mM cocktail). Bicinchoninic acid assay (BCA) method was used to determine protein concentration. Equal amounts of protein were loaded and resolved by electrophoresis on a 10 % polyacrylamide gel. The semi-dry method was used to transfer proteins onto a PVDF membrane which was then blocked with 5 % non-fat dry milk overnight. After TBST washing, membrane was incubated for 2 h with primary antibodies and then washed again with TBST before incubation with secondary antibodies for 2 h. Then X-ray autoradiography was performed and the gray scale images were analysed.

The article "Glycol chitosan incorporated retinoic acid chlorochalcone (RACC) nanoparticles in the treatment of Osteosarcoma" was retracted in 2020. Reasons: results that could not be reproduced; duplicated images; concerns about the images.

### Flow cytometric analysis

Identification of apoptosis and necrosis in osteosarcoma cells was performed by propidium iodide and FITC-annexin V reagents respectively. Treatment of cells with various concentrations of RACC-incorporated GC nanoparticles for 24 h was followed by washing with PBS. After suspension in binding buffer (10 mM HEPES pH 7.4, 150 mM NaCl, 5 mM KCl, 1 mM MgCl_2_, and 1.8 mM CaCl_2_) containing FITC annexin V (1 μg/mL) the pellets were incubated for 20 minutes. Then PI (10 μg/mL) was added to stain necrotic cells under dark conditions and incubation was continued for 10 minutes more. FAC Scan flow cytometer (Becton Dickenson Biosciences, San Jose, CA, USA) was used to analyse the cells immediately.

### Detection of Single-Strand DNA (ssDNA)

In a 96-multiwell plate, 10000 cells/well were seeded and incubated with the RACC-incorporated GC nanoparticles. The cells were then fixed with 80 % methanol for 30 minutes. The plates were dried and incubated with formaldehyde for 10 min at room temperature followed by 10 min at 75 °C, and then at 4 °C for 5 min. With 3 % non-fat dry milk cells were incubated for 1 h followed by incubation with the antibody mixture (containing a primary monoclonal antibody to ssDNA and horseradish peroxidase-labeled secondary antibody) for 30 min. The addition of 2-2’-azino-bis[3-ethylbenziazoline-6-sulfonic acid] solution permitted the reading of the plates at 405 nm in a standard microtiter reader. As positive control ssDNA and as negative control necrotic cells obtained by hyperthermia were used.

### Immunocytochemistry for Has

Onto the chamber slides (BD Biosciences, Mountain View, CA, USA) 2.5 × 10^6^ MG-63 cells were seeded and allowed to stick to the bottom. The cells were then incubated with various concentrations of RACC for 24 h and subjected to Has1 and Has3 immunocytochemistry. The antibodies against Has1 and Has3 were raised in rabbits by subcutaneous injection of the synthetic peptides.

### Motility and matrigel invasion assays

Transwell motility chambers were used to analyse cell migration and invasion. For this, the 8-mm pore diameter transwell motility chambers (Corning) were coated with matrigel (BD Biosciences) on undesurfaces. Into the upper chamber, 2 × 10^6^ cells were plated in serum-free culture medium and the lower chamber was filled with medium containing 10 % FBS. The plates were incubated for 24 hours at 37 °C. After incubation the upper surface of the compartment was cleaned. The inserts after methanol fixing were stained with crystal violet solution (0.5 %) followed by microscopic examination. The 5 areas were randomly selected and the cells were calculated. Experiments were performed in triplicates.

The article "Glycol chitosan incorporated retinoic acid chlorochalcone (RACC) nanoparticles in the treatment of Osteosarcoma" was retracted in 2020. Reasons: results that could not be reproduced; duplicated images; concerns about the images.

### Effects of RACC in vivo

The dorsal flank of 5-week-old C3H/He male mice were transfected with MG-63 cells (2.5 × 10^6^) suspended in 200 ml of serum-free DMEM. After 14 days of in vivo growth small tumours (0.6–1.2 cm in diameter) were observed. The mice were then randomly assigned into two groups with 10 each. The mice in RACC group received 15 mg RACC with 100 ml of 0.4 % CMC solution intraperitoneally daily whereas the mice in control group were given same amount of 0.4 % CMC solution. Twenty days after the treatment, the mice were sacrificed, and their tumours were excised and analysed for tumour wet weight and number of metastatic colonies. All animal experiments were performed in accordance with the National Cancer Research Institute (2010) Guidelines for the welfare and use of animals in cancer research and under approval of the institutional animal ethics committee.

### HA staining for cells and tissues

The hyaluronic acid binding protein (HABP; Seikagaku, Tokyo, Japan) was used to examine the accumulation of hyaluronan in cells and in vivo tissues with or without RACC. MG-63 cells were distributed onto chamber slides (BD Biosciences) and allowed to adhere to the bottom. The cells were then incubated with various concentrations of RACC with or without exogenous 200 mg ml^−1^ of HA for 72 h. After HABP staining, the cells and local tumours were incubated with a 2.0 mg ml^−1^ biotinylated HABP probe for 1 h at room temperature. Streptavidin-peroxidase reagents (Nichirei, Tokyo, Japan) and diaminobenzidine-containing substrate solution (Nichirei) were used to analyse b-HABP binding.

### HA quantification

MG-63 cells were incubated with or without 20 μM RACC for 6, 12, and 24 h. The cells were incubated for 10 min at 37 °C with trypsin-EDTA followed by PBS wash to remove the cell-surface-associated HA. The cells were then placed in Protease K solution (0.15 M Tris–HCl, pH 7.5, 0.15 M NaCl, 10 mM CaCl_2_, and 5 mM deferoxamine mesylate containing 20 units of protease K) and incubated for 2 h at 55 °C. For inactivation of the protease activity samples were heated at 100 °C for 20 min and centrifuged at 12 000 g for 45 min at 4 °C. The supernatants were analysed for HA concentrations using a sandwich enzyme-linked immunosorbent assay.

### Statistical analysis

The in vitro quantitative experiments were performed in triplicates, and analysis of variance followed by Bonferroni-Dunn post-hoc test was used to assess differences between means. Student’s t-test was used for statistical comparisons between the two groups.

The article "Glycol chitosan incorporated retinoic acid chlorochalcone (RACC) nanoparticles in the treatment of Osteosarcoma" was retracted in 2020. Reasons: results that could not be reproduced; duplicated images; concerns about the images.

## Abbreviations

GC: Glycol chitosan
RACC: Retinoic acid chlorochalcone
OD: Optical density
PI: Propidium iodide
